RETRACTED

# Benefits and Barriers of Holistic Nursing Training by High-Fidelity Simulation in Obstetrics

**DOI:** 10.1155/2022/1848849

**Published:** 2022-06-28

**Authors:** Wenxi Zhang, Inna Lozynska, Wei Li, Nana Cai, Hongmin Yang

**Affiliations:** ^1^Sanquan College of Xinxiang Medical University, Henan, China; ^2^Sumy National Agrarian University, Sumy, Ukraine; ^3^Henan Institute of Science and Technology, Xinxiang, China

## Abstract

**Background:**

With **t**he technology of high-fidelity simulates developed, the clinical education route has changed. The nursing school pays attention on the use of high-fidelity simulations in nursing education. However, in China, only a few schools can afford the expensive teaching tools, including SimMom 3G and virtual reality (VR) devices, which also focus on “holistic nursing simulation.”

**Objective:**

To explore the evaluation and development of a holistic nursing simulation session for nursing students based on an integrated nursing approach in obstetrics.

**Methods:**

This study was based in a rich Chinese nursing school under the medical university that value nursing education. This study is founded on 147 third-year nursing students in obstetrics classes. After the simulation teaching, the teaching effect of the questionnaire was investigated, and the total number of questionnaires was 124 students.

**Results:**

Students agreed that the holistic nursing simulation cultivated humanistic care literacy, clinical practice ability, and clinical thinking ability; enhanced teamwork ability; and reinforced professional knowledge.

**Conclusion:**

This simulation teaching method helps to cultivate students' enthusiasm and initiative and fosters their self-learning ability.

## 1. Introduction

With the rapid changes in advanced technologies in clinical nursing education, the application of simulation technology as a teaching tool has led to the application of simulation technology. Therefore, innovative approaches are needed to prepare nurses to keep up with new technologies for modern clinical practice. In the United States, simulation is widely used in multiple disciplines to train and educate people, not only in healthcare but also in aviation and the military. In the clinical nursing session, high-fidelity simulation and 3-dimensional (3D) virtual reality (VR) device can be used as a strategy used to experience realistic clinic situations [1].

Nursing skills are important, especially when treating Panenet requires comprehensive care. This simulation combines two parts, comprehensive care and technology, for nursing procedures. Simulation provides nurse students opportunities to practice skills and knowledge while using simulators, standardized patients, and virtual settings. Holistic nursing refers to patient-centered care, meaning the nurse should treat the patient as a unified human being [2].

RETRACTED

Chinese nursing schools used simulation around the beginning of the 1990s. In China, nursing simulation is practiced at various levels of fidelity: human patient simulators (nursing classmates), computer-assisted simulation (SimMan, SimBaby, SimMom), standardized patients (SP), and partial simulation (bottoms, arms, pelvis etc.); now some schools have VR devices under the different clinical scenarios. The computer-assisted simulation is an example of a high-fidelity simulator, which presents vital signs such as BP/HR/P/RR and appropriate responses to medications and other treatments.

A holistic approach to care based on simulation-based learning (SBL) may help improve the safety and quality of patient-centered care. The simulation began as a new supplement to traditional clinical experiences integrated into the curriculum in the 1960s in America [3]. It has recently been cited by the American National Council of State Boards of Nursing (NCSBN) as an effective replacement for the clinical hours in prelicensure that nurses education [4]. By the conclusion of this landmark simulation study of NCSBN, many nursing programs tend to increase the use of simulation.

The term was cited zero times in the literature search for the “holistic care simulation” study. However, in 2018, Walker and Avant advanced the development of model cases, including the defining attributes of overall nursing through simulation. Careful study of the cases is important to distinguish whether the term “holistic care simulation” is used appropriately. While care tends to classify many of the ideas in care as a whole, analyzing cases using Avant and Walker concepts will help clarify the correct holistic care simulation concept.

In this study, a case from Walker and Avant's 2018 publication was used to train Chinese nursing students, focusing on the simulation's teaching outcome. The study results will help students and teachers understand the holistic nursing simulation process from different perspectives, thus designing improved simulation training programs or cases.

## 2. Methodology

During this study, all participating students used the same following model case as Wendy (below) in the holistic nursing simulation. This case, which consisted of nine steps, is illustrated in Figure 1.

### 2.1. Model Case

Step 1. Wendy is a 3rd year nursing student who attends a holistic nursing simulation session in obstetrics class. The lecture about normal delivery was given to the class a month ahead of time for preparation in the simulation class. The holistic nursing simulation should aim patient's physical, psychosocial, spiritual, and cognitive care.

RETRACTED

Step 2. When Wendy arrives at the simulation center in the following case, she will accept that SimMom (named Pearson) will be used in this normal labor. Patient information is as follows: Mrs. Pearson, 28 years, G1P0 (Pregnancy 1 gives birth to 0), 39 +6 weeks fetus. At 9 o'clock in the cervix, the fetal head was S 1, the membrane was ruptured naturally, the amniotic fluid was clear, and the fetal heart rate was 120 beats/min after uterine contractions. Contractions are 2 to 4 minutes apart and last 30 to 45 seconds. The mother sweats at an older age, her face is tired, and when the contractions occur, the mother wants to fall asleep and the waist is sore, but there is no feeling of defecation. After 35 minutes, the maternal uterine contraction has a feeling of defecation, the anus is loose, and the fetal head is exposed. The fetal heart rate is 115 beats per minute, the interval between uterine contractions is 2 to 3 minutes, and the duration is 30 to 50 seconds. Wendy's assignment is to cooperate with the doctor to complete the delivery operation according to the situation.

Step 3. Wendy has nursing interventions in the nursing process with Pearson by first performing a thorough assessment, such as mental state, blood pressure, contractions, fetal heart, fetal head drop and extubation, and whether there is urine before delivery bed. Other students set measurable goals and nursing interventions aimed at Pearson's physical and emotional symptoms. Based on Maslow's hierarchy of needs, Wendy prioritizes nursing care in the pathophysiology and psychology of Pearson's signs.

Step 4. As a midwife, Wendy should wear a mask, hat and gloves, clean her hands, and wear a surgical gown; other classmates prepare the equipment, and sterile package, neonatal radiation table, and neonatal room rescue items are ready; make sure the environment is quiet, clean, keep warm, and protect the privacy for Mrs. Pearson. Carry the material to the delivery bed, and check and explain clearly in place; the puerpera accept cooperation. Help Mrs. Pearson take comfortable correct position, and expose abdomen and perineum.

Step 5. Wendy gives supportive care: communication with Mrs. Pearson, even the dietary support. Other classes evaluate the fetal heart every 5 to 10 minutes or several uterine contractions interval auscultation of the fetal heart. Perform perineal disinfection according to the nursing routine, and lay disinfection sheets according to the needs of different delivery positions. Timely protect perineum, assist fetal head delivery and natural shoulder delivery method, and give maternal support and encouragement all the time.

RETRACTED

Step 6. After the labor process, Wendy uses the VR device to experience neonatal care: give a blanket to keep warm, and clean the respiratory tract, neonatal assessment, early contact, early sucking, etc., waiting for the disappearance of umbilical cord pulsation or the umbilical cord after placenta delivery.

Step 7. Throughout the experience, Wendy communicates with Mrs. Pearson (SP played) about her and the newborn baby's condition. Ask the satisfaction and advice in the process, ask if she needs rest and leave her alone, and then check her condition several times after. Record all data in this normal delivery and end the cases.

Step 8. After the simulation, Wendy with classmates does debriefing, led by fully trained simulation teachers. Wendy and other students expressed the feeling that they were required to synthesize what they had learned in this normal delivery case.

Step 9. Finally, all participating students watch a video recording in the debriefing room and write a feedback focus on their performances related to each assignment under the holistic nursing approach.

### 2.2. Data Analysis

We provided a questionnaire to the participants to generate research data and specify the questions in Chinese. The quantitative data were analyzed in SPSS version 24 software.

The reliability of the questionnaire was evaluated with Cronbach's alpha. First, report the survey results of closed-ended questions and then discuss the answers to the questions raised in the open reply part of the questionnaire. In each table, the maximum response percentage for each question becomes thicker.

## 3. Results

The questionnaire was designed to examine the participants' views on whether they found it a beneficial and simulation lesson. Cronbach's alpha was 0.924, representing a high level of internal consistency [5]. From the total of 147 participating students, 124 responses were collected. The students agreed that the holistic nursing simulation cultivated humanistic care literacy, clinical practice ability, and clinical thinking ability; enhanced teamwork ability; and reinforced professional knowledge. The breakdown of the responses is given in Tables 1–5.

### 3.1. Open-Ended Questions

After the questionnaire's investigation, the participants were invited to offer advice about the simulation session as a whole as well as about this lesson. The participants commented on the simulation's several aspects. The following were stated from the simulation session students, including positive and negative feedback:

“Very realistic.”

“It was helpful to learn while using my own initiative.”

RETRACTED

“It was a very good way to study, especially combined with traditional teaching.” “Learning about critical thinking in a practical environment was enjoyed.”

“Hands on so many demonstrations.”

“Teachers had rich clinical experience and offered a lot of experience for us.”

“It needs to be improved to make it more realistic.”

“ Hope we can do more cases in other subjects.”

“ The teacher should give hints when I forget what to do.”

“We should have more simulation lessons and longer time in each lesson.”

“If there were more simulators in the simulation lab, it would solve this problem.”

The main issues raised by respondents to improve the simulation process are related to the size of the participant group during the simulation activity. Many respondents called for fewer students in the group around the bed working in manikin so that they could get more hands on the experience for future sessions. Other respondents said that a variety of examples should be carried out to gain more knowledge.

## 4. Discussion

This is a unique study that focuses on holistic nursing simulation in obstetrics. As the result, the simulation greatly promoted individual ability, and it was positive for the participation in the new learning approach. The simulation deepened the understanding of the nursing process's assessment, execution, and evaluation. As an innovative learning method, holistic simulation allows students to repeatedly practice personal and comprehensive nursing skills in an experiential way [6].

During this model case simulation, the students strongly agreed with most of the questions regarding improving their ability. This shows the benefits of holistic nursing simulation. However, the technique has several limitations that we need to discuss and revise in the future. In the section on professional knowledge and skills (Table 1), 20.16% of students responded that they could not apply basic nursing care proficiently, and 21.78% expressed an inability to comprehensively apply various specialist nursing interventions. Holistic nursing simulation tests students' skill development in every professional aspect. Therefore, many students felt that their nursing interventions were poor during those parts of the demonstration in which they were less proficient.

Clinical strategy is essential for mature clinical nurses. According to Table 2, approximately 4% of students thought that this simulation would not help them avoid the mistakes of others, and 5.56% were unable to respond quickly when the patient's situation changed. Unlike a previous study [7] that involved simulation training, our questionnaire obtained individualized responses from each student. Most students responded that they could recognize their own mistakes and react quickly. Students need adequate orientation on different simulation equipment's use prior to the class itself, as a simulation is a new learning approach. Simulation-assisted nurses' experience may not exactly replicate real clinical settings. The students' learning experience is contingent on many factors [7], such as how well the simulation is organized and how typical the simulation scenario is. Faculty's teaching style also affects the outcomes and learning perception. In the section on developing professional and critical thinking (Table 5), a single student responded that they could not conduct self-criticism and self-assessment frequently or proactively offer constructive opinions. This student may have had low self-esteem or encountered an unexpected event during the simulation.

RETRACTED

In most cases, simulation-assisted learning provides a very realistic patient and an ideal learning context, but it is still far more complex than actual clinical settings. Therefore, if possible, students still need to practice their skills in actual clinical settings: simulation cannot completely replace clinical practice. For specific practice content elements rarely encountered in clinical settings, however, simulation is an ideal alternative [8]. Unlike traditional teaching methods, simulation demands students' self-oriented learning. Most of this study's results confirm the overall simulation's effectiveness. It is expected that this paper will provide nurse educators guide to aid the future development of learning strategies and interactive and innovative teaching.

However, this study also has some shortcomings. This study is only applied in obstetrics and whether other departments can also achieve better results. In addition, the sample size is small, and the training content focuses on clinical needs. The training of higher-level obstetric nurses needs to be further explored, and a larger sample is still needed to further improve the training plan.

## 5. Conclusion

The simulation teaching method not only improves the ability of teachers, but also helps to cultivate students' initiative and enthusiasm and promotes independent learning ability.

## Figures and Tables

**Figure 1:** Step-by-step process of model case.

**Table 1:** Professional knowledge and skills.

Professional knowledge and skills	SA	A	U	D	SD
I took the initiative to make a patient nursing assessment	52.42%	29.84%	16.13%	1.61%	0%
I promptly checked for changes in the patient's condition and made appropriate nursing interventions	43.55%	36.29%	18.55%	1.61%	0%
I applied basic nursing care proficiently	37.1%	42.74%	15.32%	4.84%	0%
I comprehensively applied various specialist nursing interventions	36.29%	41.94%	16.13%	5.65%	0%

Key: SA: strongly agree; A: agree; U: unsure; D: disagree; SD: strongly disagree.

RETRACTED

**Table 2:** Clinical strategy.

Clinical strategy	SA	A	N	D	SD
The simulation process was helpful to demonstrate clinical decision-making skills	61.29%	22.58%	15.32%	0.81%	0%
The simulation could help me avoid the mistakes of others	38.71%	43.55%	13.71%	4.03%	0%
I had a sense of accomplishment when the patient got better in the simulation session	74.19%	12.9%	12.1%	0.81%	0%
I gained self-confidence in the decision-making of clinical practice	45.16%	40.32%	13.71%	0.81%	0%
I realized the importance of theoretical learning in the simulation process	55.65%	22.58%	20.16%	1.61%	0%
I responded quickly when the patient's situation changed	38.71%	37.9%	17.74%	5.65%	0%

**Table 3:** Teamwork.

Teamwork	SA	A	N	D	SD
I understood the work assigned to my team	62.1%	18.55%	16.13%	3.23%	0%
I tried to encourage cooperation among team members in the simulation session	66.13%	16.94%	16.94%	0%	0%
The team members helped and supported each other	68.55%	13.71%	16.94%	0.81%	0%
I tried my best to achieve the goals	68.55%	15.32%	14.52%	0.81%	0.81%

**Table 4:** Communication.

Communication	SA	A	N	D	SD
1. Spontaneously inquiring about psychological health of the patient	50.81%	31.45%	16.94%	0.81%	0%
2. Communicating with team members frankly	66.13%	13.71%	20.16%	0%	0%
3. Asking for teachers' help proactively	54.84%	25.81%	16.94%	2.42%	0%

**Table 5:** Development of professional and critical thinking.

Development of professional and critical thinking	SA	A	N	D	SD
Gradually adapt to the clinical role through the guidance of the teacher	51.61%	32.26%	13.71%	2.42%	0%
Conduct self-criticism and self-assessment frequently	58.87%	23.39%	13.71%	3.23%	0.81%
Can find and solve problems continuously	55.65%	28.23%	15.32%	0.81%	0%
Think positively when encountering problems	54.84%	25.81%	17.74%	1.61%	0%
Proactively offer constructive opinions	39.52%	40.32%	16.13%	3.23%	0.81%
Improve self-ability though simulation practice	53.23%	29.03%	14.52%	3.23%	0%

## Data Availability

The datasets used and analyzed during the current study are available from the corresponding author upon reasonable request.
